This article has been retracted.

# *cyclo*-Tetrakis(μ_2_-3-sulfidopropyl-κ^3^ *C* ^1^,*S*:*S*)tetrakis[chloridocobalt(III)]

**DOI:** 10.1107/S1600536811013067

**Published:** 2011-04-13

**Authors:** Shafique Ahmad Awan, M. Nawaz Tahir, Iram Khushi Muhammad, Saeed Ahmad, Muhammad Ilyas Tariq

**Affiliations:** a PAEC, PO Box # 1114, Islamabad GPO 44000, Pakistan; b Department of Physics, University of Sargodha, Sargodha, Pakistan; c Department of Chemistry, University of Engineering and Technology, Lahore 54890, Pakistan; d Department of Chemistry, University of Sargodha, Sargodha, Pakistan

## Abstract

In the centrosymmetric title compound, [Co_4_Cl_4_(C_3_H_6_S)]_4_], the two independent Co^III^ ions are each coordinated in a distorted tetra­hedral geometry by one C, one Cl and two S atoms. The mol­ecules are stabilized by C—H⋯Cl hydrogen bonds. In the crystal, inter­molecular C—H⋯Cl and C—H⋯S hydrogen bonds with *R*_2_^2^(8), *R*_4_^2^(8) and *R*_2_^2^(6) ring motifs generate a polymeric network.

## Related literature

For related background see: Shahid *et al.* (2009 ▶); Altaf *et al.* (2010 ▶). For related structures, see: Duan *et al.* (1997 ▶); Tremel *et al.* (1992 ▶). For graph-set notation, see: Bernstein *et al.* (1995 ▶).

## Experimental

### 

#### Crystal data

[Co_4_Cl_4_(C_3_H_6_S)]_4_]
*M* *_r_* = 674.07
Monoclinic,
*a* = 23.6135 (12) Å
*b* = 7.8465 (3) Å
*c* = 16.8693 (9) Å
β = 130.440 (4)°
*V* = 2378.9 (2) Å^3^
*Z* = 4
Mo *K*α radiation
μ = 3.54 mm^−1^
*T* = 296 K
0.24 × 0.16 × 0.14 mm

#### Data collection

Bruker Kappa APEXII CCD diffractometer
Absorption correction: multi-scan (*SADABS*; Bruker, 2005 ▶) *T*_min_ = 0.675, *T*_max_ = 0.683
13736 measured reflections
2152 independent reflections
1782 reflections with *I* > 2σ(*I*)
*R*_int_ = 0.058

#### Refinement

*R*[*F* ^2^ > 2σ(*F* ^2^)] = 0.041
*wR*(*F* ^2^) = 0.125
*S* = 1.04
2152 reflections
109 parameters
H-atom parameters constrained
Δρ_max_ = 0.70 e Å^−3^
Δρ_min_ = −0.62 e Å^−3^

### 

Data collection: *APEX2* (Bruker, 2009 ▶); cell refinement: *SAINT* (Bruker, 2009 ▶); data reduction: *SAINT*; program(s) used to solve structure: *SHELXS97* (Sheldrick, 2008 ▶); program(s) used to refine structure: *SHELXL97* (Sheldrick, 2008 ▶); molecular graphics: *ORTEPIII* (Burnett & Johnson, 1996 ▶), *ORTEP-3 for Windows* (Farrugia, 1997 ▶) and *PLATON* (Spek, 2009 ▶); software used to prepare material for publication: *WinGX* (Farrugia, 1999 ▶) and *PLATON*.

## Supplementary Material

Crystal structure: contains datablocks global, I. DOI: 10.1107/S1600536811013067/si2349sup1.cif

Structure factors: contains datablocks I. DOI: 10.1107/S1600536811013067/si2349Isup2.hkl

Additional supplementary materials:  crystallographic information; 3D view; checkCIF report

## Figures and Tables

**Table 1:** Selected bond lengths (Å)

Co1—Cl1	2.228 (2)
Co1—S1	2.3570 (17)
Co1—S2	2.318 (2)
Co1—C3	2.038 (6)
Co2—Cl2	2.236 (3)
Co2—S1	2.305 (2)
Co2—S2^i^	2.3648 (16)
Co2—C6^i^	2.051 (6)
S1—C1	1.826 (7)
S2—C4	1.837 (8)

Symmetry code: (i) .

**Table 2:** Hydrogen-bond geometry (Å, °)

*D*—H⋯*A*	*D*—H	H⋯*A*	*D*⋯*A*	*D*—H⋯*A*
C3—H3*A*⋯S2^ii^	0.97	2.57	3.539 (8)	175
C3—H3*B*⋯Cl2^iii^	0.97	2.74	3.512 (7)	138
C3—H3*B*⋯Cl2^iv^	0.97	2.81	3.412 (6)	121
C6—H6*A*⋯Cl1^i^	0.97	2.62	3.379 (7)	135
C6—H6*B*⋯Cl1^v^	0.97	2.48	3.343 (7)	148

Symmetry codes: (i) ; (ii) ; (iii) ; (iv) ; (v) .

## supplementary crystallographic information

### Comment

Recently, we have reported the crystal structure of zinc(II) and mercury(II) complexes of pyrrolidinedithiocarbamate (PDTC) (Shahid *et al.*, 2009) & (Altaf, *et al.*, 2010). In the present study, we attempted to prepare a cobalt(II) complex with PDTC, but surprisingly the title compound (I, Fig. 1) was isolated, the crystal structure of which is being presented.

The crystal structure of (II) i.e, tetranuclear molecular square[Co(HL)]_4_^4+^ [H_2_L = tetra(2-pyridyl)thiocarbazone] (Duan *et al.*, 1997) and (III) *i.e.*, bis(tetraethylammonium) hexakis(µ_2_-phenylthiolato)-tetrachloro-tetra -cobalt acetonitrile solvate (Tremel *et al.*, 1992) have been published which are related to the title compound (I).

The crystal structure of the title compound (I) is centrosymmetric. The coordination around two independent Co^iii^ ions is distorted tetrahedral from one C, Cl and two S-atoms. The range of Co—C [2.038 (6)–2.051 (6) Å] is shorter compared to Co—S [2.305 (2)–2.3648 (16) Å]. The Co—Cl bonds have values of 2.228 (2) and 2.236 (2) Å. The important bond distances are given in Table 1. The molecules are stabilized in the form of a polymeric network due to C—H···Cl and C—H···S intermolecular H-bonds (Table 2) forming *R*_2_^2^(8), *R*_4_^2^(8) and *R*_2_^2^(6) ring motifs (Bernstein *et al.*, 1995).

### Experimental

The title compound was prepared by adding two equivalents of ammonium pyrrolidinedithiocarbamate (PDTC) in 15 ml methanol to a solution of CoCl_2_.6H_2_O in 10 ml methanol. The addition of PDTC in the pink colored metal ion solution resulted in the formation of green precipitates immediately. After stirring for half an hour, the precipitates were filtered off and dried. The blackish brown crystals of the title compound (I) were prepared by dissolving 0.03 g precipitates in 3 ml DMSO on heating in a vial and then cooling the resulting solution at room temperature.

### Refinement

The H-atoms were positioned geometrically (C–H = 0.97 Å) and were included in the refinement in the riding model approximation, with *U*_iso_(H) = *xU*_eq_(C), where *x* = 1.2 for all H-atoms.

### Crystal data

**Table:**

[Co_4_Cl_4_(C_3_H_6_S)]_4_]	*F*(000) = 1344
*M**_r_* = 674.07	*D*_x_ = 1.882 Mg m^−^^3^
Monoclinic, *C*2/*c*	Mo *K*α radiation, λ = 0.71073 Å
Hall symbol: -C 2yc	Cell parameters from 1782 reflections
*a* = 23.6135 (12) Å	θ = 2.3–25.2°
*b* = 7.8465 (3) Å	µ = 3.54 mm^−^^1^
*c* = 16.8693 (9) Å	*T* = 296 K
β = 130.440 (4)°	Prisms, white
*V* = 2378.9 (2) Å^3^	0.24 × 0.16 × 0.14 mm
*Z* = 4	

### Data collection

**Table:**

Bruker Kappa APEXII CCD diffractometer	2152 independent reflections
Radiation source: fine-focus sealed tube	1782 reflections with *I* > 2σ(*I*)
graphite	*R*_int_ = 0.058
Detector resolution: 8.10 pixels mm^-1^	θ_max_ = 25.2°, θ_min_ = 2.3°
ω scans	*h* = −28→28
Absorption correction: multi-scan (*SADABS*; Bruker, 2005)	*k* = −9→8
*T*_min_ = 0.675, *T*_max_ = 0.683	*l* = −20→20
13736 measured reflections	

### Refinement

**Table:**

Refinement on *F*^2^	Primary atom site location: structure-invariant direct methods
Least-squares matrix: full	Secondary atom site location: difference Fourier map
*R*[*F*^2^ > 2σ(*F*^2^)] = 0.041	Hydrogen site location: inferred from neighbouring sites
*wR*(*F*^2^) = 0.125	H-atom parameters constrained
*S* = 1.04	*w* = 1/[σ^2^(*F*_o_^2^) + (0.0653*P*)^2^ + 15.5359*P*] where *P* = (*F*_o_^2^ + 2*F*_c_^2^)/3
2152 reflections	(Δ/σ)_max_ < 0.001
109 parameters	Δρ_max_ = 0.70 e Å^−^^3^
0 restraints	Δρ_min_ = −0.62 e Å^−^^3^

### Special details

**Table:**

Geometry. Bond distances, angles *etc*. have been calculated using the rounded fractional coordinates. All su's are estimated from the variances of the (full) variance-covariance matrix. The cell e.s.d.'s are taken into account in the estimation of distances, angles and torsion angles
Refinement. Refinement of *F*^2^ against ALL reflections. The weighted *R*-factor *wR* and goodness of fit *S* are based on *F*^2^, conventional *R*-factors *R* are based on *F*, with *F* set to zero for negative *F*^2^. The threshold expression of *F*^2^ > σ(*F*^2^) is used only for calculating *R*-factors(gt) *etc*. and is not relevant to the choice of reflections for refinement. *R*-factors based on *F*^2^ are statistically about twice as large as those based on *F*, and *R*- factors based on ALL data will be even larger.

### Fractional atomic coordinates and isotropic or equivalent isotropic displacement parameters (Å^2^)

**Table:**

	*x*	*y*	*z*	*U*_iso_*/*U*_eq_	
Co1	0.17597 (4)	−0.17781 (9)	0.30876 (5)	0.0323 (2)	
Co2	0.14629 (4)	−0.12119 (9)	0.50575 (5)	0.0336 (2)	
Cl1	0.09923 (9)	−0.3988 (2)	0.25283 (12)	0.0555 (5)	
Cl2	0.07469 (11)	0.0860 (3)	0.49043 (15)	0.0694 (7)	
S1	0.21157 (8)	−0.0272 (2)	0.45587 (11)	0.0460 (4)	
S2	0.28224 (8)	−0.2358 (2)	0.33225 (11)	0.0481 (5)	
C1	0.1631 (4)	0.1666 (8)	0.3814 (5)	0.066 (3)	
C2	0.0959 (4)	0.1316 (9)	0.2708 (5)	0.061 (2)	
C3	0.1163 (3)	0.0287 (7)	0.2182 (4)	0.0362 (17)	
C4	0.3356 (4)	−0.0372 (9)	0.3904 (6)	0.064 (3)	
C5	0.4140 (4)	−0.0689 (10)	0.4862 (6)	0.065 (3)	
C6	0.4164 (3)	−0.1622 (7)	0.5638 (4)	0.0417 (17)	
H1A	0.14799	0.22914	0.41469	0.0787*	
H1B	0.19711	0.23811	0.38263	0.0787*	
H2A	0.05934	0.07031	0.26878	0.0733*	
H2B	0.07391	0.23855	0.23404	0.0733*	
H3A	0.14572	0.09690	0.20863	0.0435*	
H3B	0.07165	−0.00820	0.15024	0.0435*	
H4A	0.33533	0.02242	0.33979	0.0769*	
H4B	0.31166	0.03559	0.40757	0.0769*	
H5A	0.43922	−0.13460	0.46849	0.0783*	
H5B	0.43980	0.03894	0.51537	0.0783*	
H6A	0.39644	−0.09200	0.58805	0.0502*	
H6B	0.46733	−0.19168	0.62322	0.0502*	

### Atomic displacement parameters (Å^2^)

**Table:**

	*U*^11^	*U*^22^	*U*^33^	*U*^12^	*U*^13^	*U*^23^
Co1	0.0275 (4)	0.0399 (4)	0.0300 (4)	−0.0012 (3)	0.0189 (3)	−0.0025 (3)
Co2	0.0338 (4)	0.0373 (4)	0.0312 (4)	−0.0014 (3)	0.0217 (3)	0.0004 (3)
Cl1	0.0496 (9)	0.0537 (9)	0.0545 (9)	−0.0089 (7)	0.0299 (8)	−0.0081 (7)
Cl2	0.0683 (11)	0.0733 (11)	0.0725 (12)	0.0219 (9)	0.0483 (10)	0.0114 (9)
S1	0.0485 (8)	0.0520 (8)	0.0377 (7)	−0.0099 (7)	0.0281 (7)	−0.0045 (6)
S2	0.0407 (8)	0.0667 (10)	0.0398 (8)	0.0055 (7)	0.0274 (7)	0.0030 (7)
C1	0.091 (5)	0.045 (4)	0.054 (4)	−0.010 (4)	0.044 (4)	−0.004 (3)
C2	0.066 (4)	0.047 (4)	0.056 (4)	0.003 (3)	0.033 (4)	0.008 (3)
C3	0.034 (3)	0.045 (3)	0.030 (3)	−0.003 (2)	0.021 (2)	0.005 (2)
C4	0.056 (4)	0.064 (4)	0.074 (5)	0.000 (3)	0.043 (4)	0.022 (4)
C5	0.056 (4)	0.067 (4)	0.074 (5)	−0.010 (3)	0.043 (4)	0.003 (4)
C6	0.038 (3)	0.047 (3)	0.037 (3)	−0.012 (2)	0.023 (3)	−0.005 (2)

### Geometric parameters (Å, °)

**Table:**

Co1—Cl1	2.228 (2)	C5—C6	1.469 (11)
Co1—S1	2.3570 (17)	C1—H1A	0.9700
Co1—S2	2.318 (2)	C1—H1B	0.9700
Co1—C3	2.038 (6)	C2—H2A	0.9700
Co2—Cl2	2.236 (3)	C2—H2B	0.9700
Co2—S1	2.305 (2)	C3—H3A	0.9700
Co2—S2^i^	2.3648 (16)	C3—H3B	0.9700
Co2—C6^i^	2.051 (6)	C4—H4A	0.9700
S1—C1	1.826 (7)	C4—H4B	0.9700
S2—C4	1.837 (8)	C5—H5A	0.9700
C1—C2	1.495 (10)	C5—H5B	0.9700
C2—C3	1.492 (11)	C6—H6A	0.9700
C4—C5	1.490 (13)	C6—H6B	0.9700
			
Co1···H4A^ii^	3.3200	S2···H4A^ii^	3.0500
Cl1···C3	3.473 (6)	C2···Cl2^iv^	3.570 (7)
Cl1···C6^iii^	3.343 (7)	C3···Cl1	3.473 (6)
Cl1···C6^i^	3.379 (7)	C3···S1	3.103 (5)
Cl2···C1	3.623 (11)	C3···S2	3.686 (7)
Cl2···C3^iv^	3.512 (7)	C3···C1	2.455 (9)
Cl2···C6^i^	3.492 (6)	C3···Cl2^iv^	3.512 (7)
Cl2···C3^v^	3.412 (6)	C3···Cl2^viii^	3.412 (6)
Cl2···S1	3.744 (4)	C3···S2^ix^	3.539 (8)
Cl2···C2^iv^	3.570 (7)	C6···Cl1^i^	3.379 (7)
Cl1···H4A^ii^	2.8900	C6···Cl2^i^	3.491 (6)
Cl1···H2B^vi^	2.8800	C6···Cl1^x^	3.343 (7)
Cl1···H6A^i^	2.6200	H1A···Cl2	2.9600
Cl1···H6B^iii^	2.4800	H1B···H3A	2.5900
Cl2···H1A	2.9600	H1B···S1^vii^	3.1000
Cl2···H3B^v^	2.8100	H2A···H2A^iv^	2.4400
Cl2···H3B^iv^	2.7400	H2B···Cl1^xi^	2.8800
Cl2···H5B^vii^	2.9600	H3A···H1B	2.5900
S1···Cl2	3.744 (4)	H3A···S2^ix^	2.5700
S1···S2	3.785 (3)	H3B···Cl2^iv^	2.7400
S1···C2	2.774 (7)	H3B···Cl2^viii^	2.8100
S1···C3	3.103 (5)	H4A···Co1^ix^	3.3200
S1···Co1^i^	3.8074 (16)	H4A···Cl1^ix^	2.8900
S1···S1^i^	3.773 (2)	H4A···S2^ix^	3.0500
S2···C3^ii^	3.539 (8)	H4B···S1	3.0000
S2···S1	3.785 (3)	H4B···H6A	2.5200
S2···C3	3.686 (7)	H5B···Cl2^vii^	2.9600
S1···H4B	3.0000	H6A···H4B	2.5200
S1···H1B^vii^	3.1000	H6A···Cl1^i^	2.6200
S2···H3A^ii^	2.5700	H6B···Cl1^x^	2.4800
			
Cl1—Co1—S1	118.22 (8)	C2—C1—H1B	109.00
Cl1—Co1—S2	114.37 (8)	H1A—C1—H1B	108.00
Cl1—Co1—C3	108.9 (2)	C1—C2—H2A	110.00
S1—Co1—S2	108.14 (7)	C1—C2—H2B	109.00
S1—Co1—C3	89.52 (17)	C3—C2—H2A	110.00
S2—Co1—C3	115.5 (2)	C3—C2—H2B	109.00
Cl2—Co2—S1	111.09 (9)	H2A—C2—H2B	108.00
Cl2—Co2—S2^i^	113.44 (8)	Co1—C3—H3A	110.00
Cl2—Co2—C6^i^	109.0 (2)	Co1—C3—H3B	110.00
S1—Co2—S2^i^	115.39 (8)	C2—C3—H3A	110.00
S1—Co2—C6^i^	117.5 (2)	C2—C3—H3B	110.00
S2^i^—Co2—C6^i^	88.68 (15)	H3A—C3—H3B	108.00
Co1—S1—Co2	110.96 (8)	S2—C4—H4A	109.00
Co1—S1—C1	93.3 (2)	S2—C4—H4B	109.00
Co2—S1—C1	104.4 (4)	C5—C4—H4A	109.00
Co1—S2—C4	102.5 (4)	C5—C4—H4B	109.00
Co1—S2—Co2^i^	99.94 (8)	H4A—C4—H4B	108.00
Co2^i^—S2—C4	93.3 (2)	C4—C5—H5A	110.00
S1—C1—C2	113.0 (5)	C4—C5—H5B	110.00
C1—C2—C3	110.6 (8)	C6—C5—H5A	109.00
Co1—C3—C2	108.5 (4)	C6—C5—H5B	110.00
S2—C4—C5	112.1 (5)	H5A—C5—H5B	108.00
C4—C5—C6	110.6 (9)	C5—C6—H6A	110.00
Co2^i^—C6—C5	107.9 (4)	C5—C6—H6B	110.00
S1—C1—H1A	109.00	H6A—C6—H6B	108.00
S1—C1—H1B	109.00	Co2^i^—C6—H6A	110.00
C2—C1—H1A	109.00	Co2^i^—C6—H6B	110.00
			
Cl1—Co1—S1—Co2	−7.06 (11)	S2^i^—Co2—S1—C1	−148.1 (2)
Cl1—Co1—S1—C1	−113.8 (3)	C6^i^—Co2—S1—Co1	10.1 (2)
S2—Co1—S1—Co2	−139.02 (7)	C6^i^—Co2—S1—C1	109.3 (3)
S2—Co1—S1—C1	114.2 (3)	Cl2—Co2—S2^i^—Co1^i^	−145.79 (9)
C3—Co1—S1—Co2	104.3 (2)	Cl2—Co2—S2^i^—C4^i^	110.9 (4)
C3—Co1—S1—C1	−2.5 (4)	S1—Co2—S2^i^—Co1^i^	−16.01 (8)
Cl1—Co1—S2—C4	−174.3 (3)	S1—Co2—S2^i^—C4^i^	−119.3 (4)
Cl1—Co1—S2—Co2^i^	−78.66 (7)	Cl2—Co2—C6^i^—C5^i^	−87.1 (6)
S1—Co1—S2—C4	−40.3 (3)	S1—Co2—C6^i^—C5^i^	145.4 (5)
S1—Co1—S2—Co2^i^	55.34 (7)	Co1—S1—C1—C2	30.3 (8)
C3—Co1—S2—C4	58.1 (3)	Co2—S1—C1—C2	−82.3 (7)
C3—Co1—S2—Co2^i^	153.74 (17)	Co1—S2—C4—C5	130.1 (7)
Cl1—Co1—C3—C2	95.3 (5)	Co2^i^—S2—C4—C5	29.2 (7)
S1—Co1—C3—C2	−24.5 (5)	S1—C1—C2—C3	−56.3 (9)
S2—Co1—C3—C2	−134.5 (5)	C1—C2—C3—Co1	51.0 (7)
Cl2—Co2—S1—Co1	−116.41 (8)	S2—C4—C5—C6	−57.7 (9)
Cl2—Co2—S1—C1	−17.1 (2)	C4—C5—C6—Co2^i^	54.4 (7)
S2^i^—Co2—S1—Co1	112.67 (7)		

Symmetry codes: (i) −*x*+1/2, −*y*−1/2, −*z*+1; (ii) −*x*+1/2, *y*−1/2, −*z*+1/2; (iii) *x*−1/2, −*y*−1/2, *z*−1/2; (iv) −*x*, *y*, −*z*+1/2; (v) *x*, −*y*, *z*+1/2; (vi) *x*, *y*−1, *z*; (vii) −*x*+1/2, −*y*+1/2, −*z*+1; (viii) *x*, −*y*, *z*−1/2; (ix) −*x*+1/2, *y*+1/2, −*z*+1/2; (x) *x*+1/2, −*y*−1/2, *z*+1/2; (xi) *x*, *y*+1, *z*.

### Hydrogen-bond geometry (Å, °)

**Table:**

*D*—H···*A*	*D*—H	H···*A*	*D*···*A*	*D*—H···*A*
C3—H3A···S2^ix^	0.97	2.57	3.539 (8)	175
C3—H3B···Cl2^iv^	0.97	2.74	3.512 (7)	138
C3—H3B···Cl2^viii^	0.97	2.81	3.412 (6)	121
C6—H6A···Cl1^i^	0.97	2.62	3.379 (7)	135
C6—H6B···Cl1^x^	0.97	2.48	3.343 (7)	148

Symmetry codes: (ix) −*x*+1/2, *y*+1/2, −*z*+1/2; (iv) −*x*, *y*, −*z*+1/2; (viii) *x*, −*y*, *z*−1/2; (i) −*x*+1/2, −*y*−1/2, −*z*+1; (x) *x*+1/2, −*y*−1/2, *z*+1/2.
